The article "BAP31 Promotes Proliferation, Invasion, and Metastasis of Liver Cancer Cells via Activating PI3K/AKT Pathway" was retracted in 2023. Reasons: signs of a paper mill; suspected computer-generated content; unreliable results or conclusions; concerns about the data.

# BAP31 Promotes Proliferation, Invasion, and Metastasis of Liver Cancer Cells via Activating PI3K/AKT Pathway

**DOI:** 10.1155/2022/7686728

**Published:** 2022-04-11

**Authors:** Minmin Sun, Xue Liu, Wanying Wei, Naijian Ge, Shuli Luo, Shuqun Shen, Ruiliang Ge

**Affiliations:** ^1^Department of Hepatic Surgery I, The Third Affiliated Hospital of Naval Military Medical University, Shanghai 200438, China; ^2^Department of Radioactive Intervention, The Third Affiliated Hospital of Naval Military Medical University, Shanghai 200438, China; ^3^Department of Biliary Tract Surgery II, The Third Affiliated Hospital of Naval Military Medical University, Shanghai 200438, China; ^4^Department of Outpatient, The Third Affiliated Hospital of Naval Military Medical University, Shanghai 200438, China

## Abstract

**Background:**

Many breakthroughs have been made in the clinical treatment of liver cancer, but there are still many liver cancer patients with limited treatment methods. Therefore, it is very important to find targets for early diagnosis and specific treatment of liver cancer.

**Methods:**

During the operation, 32 pairs of tumor tissues and corresponding normal liver tissues were acquired from patients. The mRNA expression was measured by qPCR. The protein expression was evaluated via Western blot. Flow cytometry assay was performed to measure the cells apoptosis. CCK-8 assay was performed to detect cell proliferation. Transwell chamber assay was applied to detect migration and invasion of SNU-449 cells.

**Results:**

BAP31 was upregulated in liver cancer tissues and cells. Knockdown of BAP31 repressed cell proliferation and enhanced cell apoptosis of liver cancer. Knockdown of BAP31 apparently upregulated apoptosis-related proteins (Bax and Caspase-3), while it downregulated antiapoptotic proteins (Bcl-2). Knockdown of BAP31 repressed migration and invasion of SNU-449 cells. In contrast with the control and si-NC group, protein expression of MMP-2 and MMP-9 was obviously lower after si-BAP31 transfection of cells. Knockdown of BAP31 repressed PI3K/AKT signaling pathways in liver cancer cells.

**Conclusion:**

Knockdown of BAP31 repressed cell proliferation, migration, and invasion in liver cancer by suppressing PI3K/AKT/mTOR signaling pathways.

## 1. Introduction

Liver cancer is an extremely frequent type of malignancy. There are approximately 850,000 new liver cancer suffers and about 810,000 deaths from liver cancer worldwide each year [1]. Due to the complex pathogenesis of cancer and the great variability of individual patients, the efficacy of currently known oncology treatment techniques is not ideal. Surgical therapy is still the preferred strategy in the clinical treatment of liver cancer, but tumor metastasis often occurs after surgery. Many patients often missed the best treatment time, so early diagnosis and targeted therapy for liver cancer is especially important. Therefore, studying the molecular mechanisms participating in the development of liver cancer is essential for new therapeutic strategies against liver cancer.

The article "BAP31 Promotes Proliferation, Invasion, and Metastasis of Liver Cancer Cells via Activating PI3K/AKT Pathway" was retracted in 2023. Reasons: signs of a paper mill; suspected computer-generated content; unreliable results or conclusions; concerns about the data.

BAP31, identified by Kim et al. [2] in 1994, belongs to a family of B cell receptor-associated proteins that selectively bind to membrane-type IgD and thus is a main factor activating B cell receptors. BAP31 also acts as a carrier protein that mediates the transport of proteins from the endoplasmic reticulum to the Golgi apparatus [3]. In addition, BAP31 is also a member of the BCL-2/BCL-XL family and can act as an apoptosis regulator that participated in the apoptosis regulation process [4]. BAP31 is upregulated in a range of cancers, such as cervical cancer [5], colorectal cancer [6], and malignant melanoma [7].

The PI3K/AKT/mTOR signaling pathway is activated in many malignancies, including colorectal cancer, ovarian cancer, and breast cancer [8]. The PI3K/AKT signaling pathway could be activated by numerous stimuli, and the PI3K/AKT complex is the main cellular molecular pathway in autophagy [9]. CD274 was found to induce the PI3K/AKT/mTOR signaling pathway to participate in numerous tumors [10]. miR-570-3p suppressed proliferation and migration of breast cancer cells and enhanced apoptosis by targeting CD274, which may be associated with inhibition of the PI3K/AKT/mTOR signaling pathway [11]. PI3K/AKT/mTOR pathway inhibitors have been effective in treating a number of cancers and have become an important target for clinical cancer therapy. However, the effects and underlying pathways of BAP31 in liver cancer are still indistinct.

In this research, knockdown of BAP31 suppressed cell proliferation, migration, and invasion in liver cancer by suppressing the PI3K/AKT/mTOR signaling pathways.

## 2. Materials and Methods

### 2.1. Patient Samples

32 pairs of tumor tissues and corresponding normal liver tissues were acquired from liver cancer patients (17 males and 15 females, from 35 to 58 years old), who came to the Third Affiliated Hospital of Naval Military Medical University for surgical treatment from May 2017 to October 2018. Patients have not received radiotherapy or chemotherapy prior to surgery. Samples are pathologically confirmed and stored at −80°C. The protocols were approved by Ethics Committee of the Third Affiliated Hospital of Naval Military Medical University. All patients who participated in the experiment signed informed consent.

### 2.2. Cells Culture

Normal liver cell lines (THLE-3) and hepatocellular carcinoma cell lines (SNU-182, SNU-423, SNU-449, and SNU-387) were obtained from the American Type Collection, USA. Cell lines were maintained in the RPMI-1640 growth medium (Procell) and 10% FBS, maintained at 37°C with 5% CO_2_. In addition, siRNA1 and siRNA2 specifically targeting BAP31 were synthesized and transfected into SNU-449 cells.

The article "BAP31 Promotes Proliferation, Invasion, and Metastasis of Liver Cancer Cells via Activating PI3K/AKT Pathway" was retracted in 2023. Reasons: signs of a paper mill; suspected computer-generated content; unreliable results or conclusions; concerns about the data.

### 2.3. RNA Isolation and Quantitative Real-Time PCR Analysis

Total tissue RNA was separated by TRIzol reagent (Corning, USA), cDNA was retrieved and mRNA expression was measured using the SYBR Premix EX Taq II kit (Takara, Japan), and the 2^−△△Ct^ method was adopted to analyse relative gene expression.

### 2.4. Western Blot

Total protein from each group was separated with RIPA reagent (Invitrogen, USA). Quantification was performed using a BCA kit. 10% SDS-PAGE was adopted to separate protein. The protein bands were transferred to a polyvinylidene difluoride (PVDF) membrane (Invitrogen, USA) by the semidry transmembrane method. Then, they were blocked using 5% skim milk for 2 h at 25. They were incubated overnight with appropriate amounts of the primary antibody (Absin, China) at 4°C. PVDF membranes were washed the next day using Tris-HCL with Tween composite buffer and then were incubated for 2 h with the secondary antibody (Cell Signaling Technology, USA). The expression of each protein was quantified by the gray scale values scanned with the Gel Imager.

### 2.5. CCK-8 Assay

The CCK-8 Kit (Dojindo, Japan) was applied to measure cell growth ability. 96-well plates were loaded with 3,000 cells per well. The cells were cultured for 72 h. The absorbance at 450 nm was detected in a specific time (24, 48, and 72 h).

### 2.6. Transwell Assay

The upper chamber was added with SNU-449 cells and serum-free medium, and the lower chamber was loaded with medium including 10% fetal bovine serum. The upper chamber shall be coated with Matrigel (BD Biosciences, USA) for invasion experiment, while the migration experiment shall be carried out without Matrigel. Then, transwell chamber was incubated at 37°C. The cells crossing the membrane were stained with crystal violet and counted after incubation for 48 h.

### 2.7. Flow Cytometry Assay

SNU-449 cells were dyed to detect cells apoptosis via FITC Annexin V/PI (Dojindo, Japan). PBS was used to wash cells, and cells were resuspended via binding buffer (10 mM HEPES/NaOH, pH 7.4; 140 mM NaCl; 2.5 mM CaCl_2_). Then, Annexin V solution and PI were added to these cells. The fluorescence intensity was measured after 1 h via flow cytometry.

### 2.8. Statistical Analysis

Analysis was conducted using SPSS 19.0 statistical software. Comparisons between groups were performed by one-way analysis of variance (ANOVA), and *P* < 0.05 was considered as statistically significant.

The article "BAP31 Promotes Proliferation, Invasion, and Metastasis of Liver Cancer Cells via Activating PI3K/AKT Pathway" was retracted in 2023. Reasons: signs of a paper mill; suspected computer-generated content; unreliable results or conclusions; concerns about the data.

## 3. Results

### 3.1. The Expression of BAP31 Raised in Liver Cancer

The mRNA expression of BAP31 was obviously higher in tumor tissues in contrast with normal tissues (Figure 1(a)). The mRNA expression of BAP31 was apparently higher in liver cancer cell lines in contrast with normal cell lines (Figure 1(b)). Protein expression of BAP31 was apparently higher in liver cancer cell lines (Figure 1(c)).

### 3.2. Knockdown of BAP31 Inhibited Cell Proliferation of Liver Cancer

In contrast with the control and si-NC group, mRNA expression of BAP31 was obviously lower after si-BAP31 transfection of cells, especially in the si2-BAP31 group (Figure 2(a)). The results of Western blot experiments are consistent. In contrast with the control and si-NC group, protein expression of BAP31 was obviously lower after si-BAP31 transfection of cells, especially in the si2-BAP31 group (Figures 2(b) and 2(c)). These results suggest that both siRNA1 and siRNA2 can effectively knockdown BAP31, especially siRNA2. Subsequently, we found that cell proliferation was obviously decreased in the si2-BAP31 group by comparison (Figures 2(d)–2(f)).

### 3.3. Knockdown of BAP31 Promoted Cell Apoptosis of Liver Cancer

In contrast with the control and si-NC group, cell apoptosis was obviously raised in the si2-BAP31 group (Figures 3(a) and 3(b)). In contrast with the control and si-NC group, Si2-BAP31 apparently upregulated apoptosis-related proteins (Bax and Caspase-3) and downregulated antiapoptotic proteins (Bcl-2) (Figures 3(c) and 3(d)).

### 3.4. Knockdown of BAP31 Suppressed Cell Migration and Invasion of Liver Cancer

In contrast with the control and si-NC group, Si2-BAP31 apparently inhibited cell migration of liver cancer (Figures 4(a) and 4(b)). In contrast with the control and si-NC group, Si2-BAP31 apparently inhibited cell invasion of liver cancer (Figures 4(c) and 4(d)). In contrast with the control and si-NC group, protein expression of MMP-2 and MMP-9 was apparently lower after si-BAP31 transfection of cells (Figures 4(e) and 4(f)).

### 3.5. BAP31 Regulated Liver Cancer via the PI3K/AKT/mTOR Signaling Pathway

In contrast with the control and si-NC group, protein expression of PI3K-AKT and mTOR was obviously lower after si-BAP31 transfection of cells (Figure 5).

## 4. Discussion

Liver cancer is currently one of the most common cancers in the world. Due to the insidious onset of liver cancer and the lack of effective clinical treatment, the five-year average survival rate is less than 10% [12]. The best treatment for liver cancer is surgical resection and liver transplantation, but the prognosis of patients with advanced liver cancer is not satisfactory due to its highly invasive nature and high susceptibility to metastasis [13]. There have been many breakthroughs in its clinical treatment, but only a minority of liver cancer patients are suitable for treatment options such as surgical resection, radiotherapy, and immune checkpoint inhibition [14]. Therefore, researchers have been working to find targets for early diagnosis and specific treatment of liver cancer.

The article "BAP31 Promotes Proliferation, Invasion, and Metastasis of Liver Cancer Cells via Activating PI3K/AKT Pathway" was retracted in 2023. Reasons: signs of a paper mill; suspected computer-generated content; unreliable results or conclusions; concerns about the data.

We are the first to explore the expression and function of BAP31 in liver cancer. Interestingly, BAP31 was upregulated in liver cancer tissues and cells. BAP31 was highly expressed in other types of cancer, such as cervical cancer [15], gastric cancer [16], and ovarian cancer [17]. BAP31 is a member of the BCL-2/BCL-XL family and can act as an apoptosis regulator involved in the apoptosis regulation process. The important characteristic of cancer is the disorder of cell proliferation and apoptosis. Based on the findings that BAP31 was upregulated in liver cancer, we hypothesized that it may affect cell proliferation in liver cancer. We knocked down BAP31 in SNU-449 cells, and the expression of BAP31 decreased obviously. Knockdown of BAP31 repressed cell proliferation and enhanced cell apoptosis of liver cancer. Apoptosis is an active process that involves the activation, expression, and regulation of a series of genes, especially Bax, Bcl-2, and Caspase-3. Knockdown of BAP31 apparently upregulated apoptosis-related proteins (Bax and Caspase-3) and downregulated antiapoptotic proteins (Bcl-2). This may be an important way for BAP31 to regulate liver cancer. In addition, knockdown of BAP31 suppressed cell migration and invasion of liver cancer. In contrast with the control and si-NC group, protein expression of MMP-2 and MMP-9 was apparently lower after si-BAP31 transfection of cells. Matrix metalloproteinase (MMPs) is a calcium-dependent, zinc-containing, structurally and functionally related endo skin enzyme that degrades the extracellular matrix [18, 19]. The above results suggest that BAP31 was involved in the regulation of liver cancer, but the exact mechanism needs to be further explored.

The development and progression of liver cancer are closely related to the activation or inhibition of certain signal transduction pathways, which regulate proliferation, differentiation, hematopoiesis, metastasis, and prognosis of liver cancer cells. The PI3K/AKT signaling pathway could be activated by numerous stimuli, and the PI3K/AKT complex is the main cellular molecular pathway in autophagy [9]. Knockout of JAK2 repressed tumor progression via enhancing apoptosis and antiproliferation by PI3K/AKT signaling pathways [20]. YARS promoted cell proliferation and invasion in gastric cancer via activating PI3K-Akt signaling [21]. We explored the relationship between BAP31 and PI3K/AKT signaling pathways. Knockdown of BAP31 inhibited the PI3K/AKT signaling pathways in liver cancer cells.

The article "BAP31 Promotes Proliferation, Invasion, and Metastasis of Liver Cancer Cells via Activating PI3K/AKT Pathway" was retracted in 2023. Reasons: signs of a paper mill; suspected computer-generated content; unreliable results or conclusions; concerns about the data.

In conclusion, knockdown of BAP31 inhibited cell proliferation, migration, and invasion in liver cancer by suppressing PI3K/AKT/mTOR signaling pathways, thus providing a potential novel therapeutic target for the diagnosis and treatment of liver cancer.

## Figures and Tables

**Figure 1:** The expression of BAP31 raised in liver cancer. (a) The mRNA expression of BAP31 higher in liver cancer tissues. (b) The mRNA expression of BAP31 higher in liver cancer cell. (c) BAP31 upregulated in liver cancer cells. *N* = 32, ^*∗*^*P* < 0.05.

**Figure 2:** `Knockdown of BAP31 repressed cell proliferation of liver cancer. (a) Si-BAP31 reduced mRNA expression of BAP31. (b)-(c). Si-BAP31 reduced protein expression of BAP31. (c) Si2-BAP31 reduced cell proliferation of SNU-449. ^*∗*^*P* < 0.05.

**Figure 3:** Knockdown of BAP31 promoted cell apoptosis of liver cancer. (a)-(b) Flow cytometry assay conducted to detect cell apoptosis. (c) Protein expression of Bax, Bcl-2, and Caspase-3 evaluated by Western blot. ^*∗*^*P* < 0.05.

**Figure 4:** Knockdown of BAP31 suppressed cell migration (a) and invasion (b) of liver cancer. (c) Protein expression measured by Western blot. ^*∗*^*P* < 0.05.

**Figure 5:** BAP31 regulated liver cancer via the PI3K/AKT/mTOR signaling pathway. ^*∗*^*P* < 0.05.

## Data Availability

The data used to support the findings of this study are available from the corresponding author upon request.
